The article "microRNA-613 exerts anti-angiogenic effect on nasopharyngeal carcinoma cells through inactivating the AKT signaling pathway by down-regulating FN1" was retracted in 2021. Reasons: duplicated images; signs of a paper mill.

# microRNA-613 exerts anti-angiogenic effect on nasopharyngeal carcinoma cells through inactivating the AKT signaling pathway by down-regulating FN1

**DOI:** 10.1042/BSR20182196

**Published:** 2019-07-10

**Authors:** Ru Gao, Qiaolei Feng, Guolin Tan

**Affiliations:** 1 Department of Otolaryngology Head and Neck Surgery, The 3rd Xiangya Hospital of Central South University, Changsha 410013, P.R. China; 2 Department of Otolaryngology Head and Neck Surgery, Hunan Aerospace Hospital, Changsha 410205, P.R. China

**Keywords:** AKT signaling pathway, FN1, Invasion, MicroRNA-613, Migration, Nasopharyngeal carcinoma

## Abstract

**Background:** Nasopharyngeal carcinoma (NPC) is a disease highly sensitive to radiotherapy with the unclear etiology. However, the specific effects of microRNA-613 (miR-613) on NPC still remain elusive. Therefore, the present study probes into the underlying mechanism of miR-613 in NPC via AKT signaling pathway by regulating Fibronectin 1 (FN1).

**Methods:** First, microarray analysis was used to screen differentially expressed genes (DEGs) and regulatory miRs associated with NPC. Next, miR-613 and FN1 expression in NPC cells was determined, followed by verification of target relationship between miR-613 and FN1. With NPC cells exposed to miR-613 mimic, si-FN1 and LY294002 (inhibitor of AKT signaling pathway), the regulatory effects of miR-613 on proliferation, apoptosis, invasion, migration and angiogenesis of NPC cells were detected with ratio of B-cell lymphoma 2/Bcl-2-associated X protein (Bcl-2/Bax), Cleaved-caspase3, matrix metallopeptidase 2 (MMP-2), MMP-9, vascular endothelial growth factor (VEGF), and cell adhesion molecule-1 (CD31) expression measured. Then, tumorigenesis and MVD were determined after Xenograft in nude mice.

**Results:** FN1 modulated by miR-613 was critical for NPC via the AKT signaling pathway. NPC cells exhibited down-regulated miR-613 and up-regulated FN1. Besides, miR-613 was verified to target FN1. Moreover, overexpressed miR-613, silenced FN1 or LY294002 treatment suppressed proliferation, invasion, migration, and angiogenesis in NPC cells, which was indicated by reduced expression of AKT, mTOR, MMP-2, MMP-9, VEGF, and CD31 as well as decreased ratio of Bcl-2/Bax and increased expression of Cleaved-caspase3. Furthermore, cell apoptosis was promoted and tumorigenesis and MVD in nude mice were inhibited with overexpression of miR-613, silenced FN1 or LY294002 treatment.

**Conclusion:** Taken together, miR-613 inhibits angiogenesis in NPC cells through inactivating FN1-dependent AKT signaling pathway.

## Background

Nasopharyngeal carcinoma (NPC), a highly malignant squamous cell carcinoma originating from epithelial cells and occurring in the nasopharynx, is associated with distant metastasis and local invasion [1]. This cancer is geographically and ethnically distributed, mostly in southern China, especially in the Cantonese area around Guangzhou [2,3]. People are very likely to suffer from NPC if they are infected with Epstein–Barr virus (EBV) or exposed to chemical carcinogens [4]. Apart from the viral environmental factors, the nonviral and environmental risk factors, encompassing undue intake of salt-preserved food and excessive tobacco smoking could also lead to NPC [5]. Various strategies have been applied to locally control NPC in patients, such as brachytherapy and stereotactic radiosurgery (SRS) after external beam radiation [6]. In spite of these treatments, over 1/3 patients still suffer from local recurrence mainly due to distant metastasis [7]. Therefore, it is in urgent need to develop new biomarkers for NPC treatment.

The article "microRNA-613 exerts anti-angiogenic effect on nasopharyngeal carcinoma cells through inactivating the AKT signaling pathway by down-regulating FN1" was retracted in 2021. Reasons: duplicated images; signs of a paper mill.

MicroRNAs (miRs) have been extensively reported to be closely involved in the developmental processes of tumors by regulating the expression of genes, including cell proliferation, migration, apoptosis, etc. [8,9]. miR-613 expression is remarkably low in human hepatocellular carcinoma (HCC) cells, and overexpression of miR-613 suppresses proliferation of HCC cells [10]. Meantime, a prior study showed that restored expression of miR-613 suppressed NPC cell invasion induced by Snail2 [11]. Moreover, miR-613 was revealed to target Fibronectin 1 (FN1) in a previous study [12]. FN1, a member belonging to the class of extracellular matrix glycoprotein, executes its functions in cellular adhesion, migration, tissue remodeling, and infection resistances [13]. High FN1 expression is responsible for metastasis, carcinogenesis, and invasion in various human carcinomas including renal cancer and colorectal cancer [14,15]. It was previously revealed that overexpressed miR-9-3p could lead to inhibited metastases and proliferation of NPC cells by reducing FN1 [13]. Furthermore, Wu et al. revealed that miR-613 modulated the AKT signaling pathway in ischemia reperfusion (I/R) [16]. A previous study has found that AKT signaling pathway regulates several cellular courses such as cell proliferation, apoptosis, and tumorigenesis, which eventually leads to NPC progression [17]. It has been revealed that the inactivation of the AKT signaling pathway could contribute to the inhibition of metastasis of NPC cells [18]. Based on these findings, it is suggested that miR-613, FN1 as well as the AKT signaling pathway may work in the development of NPC. Therefore, the present study furnishes a new potential effect of miR-613 on modulating invasion, migration, and angiogenesis of NPC cells via the AKT signaling pathway by regulating FN1.

The article "microRNA-613 exerts anti-angiogenic effect on nasopharyngeal carcinoma cells through inactivating the AKT signaling pathway by down-regulating FN1" was retracted in 2021. Reasons: duplicated images; signs of a paper mill.

## Materials and methods

### Microarray analysis

The Gene Expression Omnibus (GEO) database (https://www.ncbi.nlm.nih.gov/geo/) was employed to retrieve the microarray data related to NPC, and the ‘limma’ package in R language was used for differential analysis of the NPC-related microarray data. The differentially expressed genes (DEGs) were screened with |logFC| > 2 and *P* value < 0.05 used as the screening threshold, and the ‘pheatmap’ package was applied to construct the heatmap for DEGs. The STRING database (https://string-db.org/) was applied for gene interaction analysis, with the analysis results exported. Then, the exported analysis results were imported into the cytoscape software, and then the core degree values of 22 genes in interaction network were calculated using the statistical tool of the cytoscape software. Based on the degree values, a map of gene interaction network was constructed, with the degree values of genes labeled using different colors, the deeper color indicated the higher degree value of gene and the higher core level of gene in the interaction network. The DIANA database (http://diana.imis.athena-innovation.gr/DianaTools/index.php?r=microT_CDS/index), miRDB database (http://mirdb.org/miRDB/index.html), mirDIP database (http://ophid.utoronto.ca/mirDIP/index.jsp#r), miRSearch database (https://www.exiqon.com/miRSearch), starBase database (http://starbase.sysu.edu.cn/) and Target Scan database (http://www.targetscan.org/vert_71/) were used to retrieve the miRs that regulated FN1, with the intersection of the predicted results obtained.

### Cell culture and transfection

A total of four NPC cell lines 5-8F, CNE2, CNE1, and HONE-1 and one immortalized human nasopharyngeal epithelial cell line NP69 (American Type Culture Collection [ATCC), Manassas, VA, U.S.A.) were incubated in an incubator containing RPMI-1640 complete medium consisting of 10% fetal bovine serum (FBS), 100 μg/ml streptomycin and 100 U/ml penicillin at 37°C with 5% CO_2_ and 95% saturated humidity with the medium replaced 3–4 times per week depending on the cell growth. Cells were sub-cultured when the cell confluence reached about 80%. Reverse transcription quantitative polymerase chain reaction (RT-qPCR) was carried out to measure the level of miR-613 in each cell line in order to screen out two cell lines with the lowest miR-613 level for following cell experimentations.

CNE1 and HONE-1 cells were classified into blank (cells without any transfection), negative control (NC)-mimic (cells transfected with miR-613 NC sequence), miR-613 mimic (cells transfected with miR-613 mimic), si-NC (cells transfected with si-NC), si-FN1 (cells transfected with si-FN1), miR-613 mimic + overexpression (oe)-FN1 (cells transfected with miR-613 mimic and oe-FN1) and LY294002 groups (cells treated with 40 μmol/L LY294002, the inhibitor of the AKT signaling pathway). The target plasmids were purchased from Dharmacon (Lafayette, CO, U.S.A.). CNE1 and HONE-1 cells in logarithmic growth phase were inoculated into a 6-well plate at a density rate of 3 × 10^5^ cells/ml. When cell confluence reached 80%, cells were transfected using lipofectamine 2000 kits (Invitrogen, Carlsbad, California, U.S.A.). A total of 4 μg the target plasmid and 10 μl lipofectamine 2000 were respectively diluted using 250 μl serum-free Opti-MEM (Gibco, Carlsbad, California, U.S.A.), mixed gently, and allowed to stand for 5 min at room temperature. After that, above two mixtures were evenly mixed and allowed to stand for 20 min. The mixture was then added to the culture wells and cultured in an incubator with 5% CO_2_ at 37°C. After 4 h, with medium changed to complete medium, cells continued to be cultured for 48 h and were collected for subsequent experiments.

The article "microRNA-613 exerts anti-angiogenic effect on nasopharyngeal carcinoma cells through inactivating the AKT signaling pathway by down-regulating FN1" was retracted in 2021. Reasons: duplicated images; signs of a paper mill.

### RT-qPCR

Total RNA was extracted using Trizol (Invitrogen, Carlsbad, California, U.S.A.), followed by determination of RNA concentration using Nanodrop 2000 (Thermo Fisher Scientific, Waltham, MA, U.S.A.), Subsequently, complementary DNA (cDNA) was obtained through reverse transcription of 1 μg total RNA using PrimeScriptTM RT kit and gDNA Eraser kits (TaKaRa, Tokyo, Japan). RT-qPCR was conducted on an ABI7500 quantitative PCR instrument (Thermo Fisher Scientific, Waltham, MA, U.S.A.) using the SYBR® Premix Ex TaqTM (Tli RNaseH Plus) kits (TaKaRa, Tokyo, Japan). With glyceraldehyde-3-phosphate dehydrogenase (GAPDH) used as the internal reference of FN1 and U6 as the internal reference of miR-613, 2^−ΔΔ*C*_t_^ method was employed for calculation of the fold changes of the target genes between the experimental group and the control group. The primers (Table 1) were all provided by Shanghai GenePharma Co., Ltd. (Shanghai, China). The parallel experiments were repeated three times.

**Table 1:** The primer sequences for reverse transcription quantitative polymerase chain reaction

Gene	Primer sequence
miR-613	F: 5′-ACACTCCAGCTGGGATGGAATGTTCCTTC-3′
	R: 5′-CTCAACTGGTGTCGTGGAGTCGGCAATTCAGTTGAGAGAAACGG-3′
U6	F: 5′-CTCGCTTCGGCAGCACATATACT-3′
	R: 5′-ACGCTTCACGAATTTGCGTGTC-3′
GAPDH	F: 5′-GGCTCATGACCACAGTCCATG-3′
	R: 5′-TCAGCTCTGGGATGACCTTG-3′
FN1	F: 5′-TGATCACATGGACGCCTGC-3′
	R: 5′-GAGTCAAGCCGGACACAACG-3′

*Note*. F, forward; R, reverse.

### Western blot analysis

After 48 h of transfection, the CNE1 and HONE-1 cell line were collected, added with the lysate buffer containing phenylmethylsulfonyl (PMSF) and phosphatase inhibitors to extract the protein. After determination of the concentration of the protein, 10% sodium dodecyl sulfate (SDS) separation gel and contraction gel were prepared. The samples were mixed with the loading buffer, boiled in ice bath at 100°C for 5 min, centrifuged, and equally added to the lanes using a microinjector for protein separation using SDS-polyacrylamide gel electrophoresis (PAGE). Afterwards, the proteins were transferred onto a polyvinylidene fluoride (PVDF) membrane (Merck Millipore, MA, U.S.A.). After being incubated in 5% bovine serum albumin (BSA) for 1 h, the membrane was incubated at 4°C overnight with primary antibodies against FN1 (ab32419, 1/500), AKT (ab8805, 1/500), p-AKT (ab81283, 1/1000), mammalian target of rapamycin (mTOR, ab2732, 1/1000), p-mTOR (ab109268, 1/1000), B-cell lymphoma 2 (Bcl-2, ab32124, 1/1000), Bcl-2-associated X protein (Bax, ab32503, 1/1000), Cleaved-caspase3 (ab2302, 1/1000), cell adhesion molecule-1 (CD31, ab28364, 1/500), vascular endothelial growth factor (VEGF, ab32152, 0.02 mg/ml, 1/1000), matrix metallopeptidase 2 (MMP-2, ab37150, 1/2000), and MMP9 (ab38898, 1/1000). All these antibodies were from Abcam, Inc. (Cambridge, MA, U.S.A.). After being rinsed with Tris-buffered saline with Tween 20 (TBST) three times, the membrane was incubated with the goat anti-rabbit secondary antibody (ab205718, 1/500, Abcam, Cambridge, MA, U.S.A.) for 1 h, washed in PBS at room temperature three times (each time for 5 min), and immersed in electrochemiluminescence (ECL) reagents (Pierce, Rockford, IL, U.S.A.) at room temperature for 1 min. After removal of the liquid, the membrane was covered by food wrap, exposed by an X-ray film in the dark, developed, fixed, and observed. The Western blot images were analyzed using ImageJ2x software.

The article "microRNA-613 exerts anti-angiogenic effect on nasopharyngeal carcinoma cells through inactivating the AKT signaling pathway by down-regulating FN1" was retracted in 2021. Reasons: duplicated images; signs of a paper mill.

### Dual-luciferase reporter gene assay

In order to confirm whether miR-613 acted as transcription factor to target FN1, the 3′untranslated region (3′UTR) fragment of synthetic FN1 was inserted into the 3′UTR of pMIR-reporter luciferase gene (Beijing Huayueyang Biotechnology Co., Ltd., Beijing, China) to construct a recombinant vector FN1-wild type (Wt). The mutation site in 3′UTR fragment of FN1 was inserted into the 3′UTR of the pMIR-reporter luciferase gene (Beijing Huayueyang Biotechnology Co., Ltd.) to construct another recombinant vector FN1-mutant type (Mut). The correctly sequenced luciferase reporter plasmids FN1-Wt and FN1-Mut were respectively co-transfected with miR-613 mimic into HEK293T. With renilla luciferase used as an internal reference, cells were transfected for 48 h and lysed. The luciferase activity was measured by using the luciferase assay kit (K801-200, Biovision, Milpitas, CA, U.S.A.) and Glomax 20/20 luminometer fluorescence detector (Promega, Madison, WI, U.S.A.). The parallel experiment was repeated three times.

### 5-Ethynyl-2′-deoxyuridine assay

The 5-ethynyl-2′-deoxyuridine (EdU) solution (cell medium:EdU solution = 1000:1) was added into the cell culture plate, which was then incubated at room temperature for 2 h and washed with PBS. Then the cells were fixed with 40 g/L paraformaldehyde for 30 min, followed by incubation in glycine solution for 8 min and PBS washing. After being rinsed with PBS containing 0.5% Triton X-100 and incubated with Apollo® staining solution at room temperature avoiding exposure to light for 30 min, the cells were washed twice with methanol and PBS, respectively. Then, the cells were incubated with Hoechst 3334 reaction solution at room temperature for 20 min avoiding exposure to light. Images were captured under a fluorescence microscope. When photographed with green light at the excitation wavelength of 488 nm, the green-stained cells were proliferating cells. When photographed with purple light at the excitation wavelength of 350 nm, the blue-stained cells were total cells. With three visual fields selected, the EdU-stained cells (proliferating cells) and Hoechst 33342-stained cells (total cells) were counted. Cell proliferation rate = number of proliferating cells/number of total cells × 100%. The parallel experiment was repeated three times.

### Flow cytometry

The apoptosis of CNE1 and HONE-1 cells after 24-h culture was detected by Annexin V-fluorescein isothiocyanate (FITC)/propidium iodide (PI) double staining kits (556547, Shanghai Shuojia Biotechnology Co., Ltd., Shanghai, China). The 10 × Binding Buffer was diluted to 1 × Binding Buffer with deionized water. Cells were collected after centrifugation at 2000 rpm for 5 min at room temperature. The cells were then resuspended by precooled 1 × PBS, centrifuged at 200 rpm for 5–10 min, washed, and suspended with 300 μl 1 × Binding Buffer. After mixing with 5 μl Annexin V-FITC, the cells were incubated for 15 min at room temperature avoiding exposure to light. Finally, the cells were ice-bathed with the addition of 5 μl PI avoiding exposure to light for 5 min. The flow cytometer (Cube 6, Partec, Munster, Germany) was applied for detection of FITC at the excitation wavelength of 480 and 530 nm and PI at the excitation wavelength more than 575 nm.

### Transwell assay

After transfection for 48 h and starvation in serum-free medium for 24 h, the cells were detached, washed twice with PBS, and resuspended with serum-free Opti-MEMI medium (Invitrogen, Carlsbad, California, U.S.A.) supplemented with 10 g/L BSA, with the cell density adjusted to 3 × 10^4^ cells/ml. A 24-well plate and an 8 μm Transwell chamber (Corning Inc., Corning, NY, U.S.A.) were adopted with three chambers in each group and 100 μl cell suspension in each chamber. The basolateral chamber was incubated with the addition of 600 μl 10% RPMI-1640 medium with 5% CO_2_ at 37°C. For cell migration detection, after 48 h, cells were fixed with 4% paraformaldehyde for 30 min and the chamber was placed in 0.2% Triton X-100 solution (Sigma–Aldrich, St. Louis, MO, U.S.A.) for 15 min, and stained in 0.05% gentian violet solution for 5 min. As to cell invasion detection, 50 μl Matrigel (Sigma–Aldrich, St. Louis, MO, U.S.A.) was spread in the chamber prior to the experiment, and 48 h later, fixation and staining were performed using the above-mentioned methods. The number of stained cells was counted under an inverted microscope. Five visual fields were randomly selected for cell counting, and the number of cells was presented using mean. The parallel experiment was repeated three times.

The article "microRNA-613 exerts anti-angiogenic effect on nasopharyngeal carcinoma cells through inactivating the AKT signaling pathway by down-regulating FN1" was retracted in 2021. Reasons: duplicated images; signs of a paper mill.

### Tube formation assay

Following transfection, the cancer cells were co-cultured with human umbilical vein endothelial cell (HUVEC) (ATCC, Manassas, VA, U.S.A.). Each group was set with three duplicated wells. A total of 60 μl Matrigel was added into each well of a 96-well plate which was gently shaken to enable the Matrigel spread evenly. After the Matrigel gel was coagulated, the HUVEC (ATCC, Manassas, VA, U.S.A.) were resuspended with the supernatant of the transfected HONE-1 cells, with cell concentration adjusted to 2 × 10^5^ ml^−1^. Afterwards, the above-mentioned cell suspension (150 μl) was cultured in the 96-well plate coated with Matrigel at 37°C with 5% CO_2_ for 24 h. Then, the tube formation of HUVEC was observed under a phase contrast microscope (×100). Five visual fields were randomly selected from each group to assess the angiogenesis of HUVEC co-cultured with cancer cells in each group, which was expressed as the number of tube formation.

### Xenograft in nude mice

Forty-two 5 weeks old male BALB/c nude mice weighing 18–20 g purchased from Shanghai Laboratory Animal Center of Chinese Academy of Sciences (Shanghai, China) were housed in specific pathogen-free (SPF) environment with constant temperature of 25 ± 2°C, constant humidity of 45–50% and 12 h of dark/light cycle. The nude mice were fed with high-pressure sterilization standard laboratory diet with free access to sterile water. All nude mice were randomly classified into seven groups with six mice in each group: blank, NC-mimic, miR-613 mimic, si-NC, si-FN1, miR-613 inhibitor + si-FN1 and LY294002 groups.

The article "microRNA-613 exerts anti-angiogenic effect on nasopharyngeal carcinoma cells through inactivating the AKT signaling pathway by down-regulating FN1" was retracted in 2021. Reasons: duplicated images; signs of a paper mill.

The transfected HONE-1 cells of seven groups in exponential growth in the incubator were treated with 0.25% trypsin. The collected cells were mixed with serum-free medium to prepare single cell suspension with a concentration of 1 × 10^7^ cells/ml. Subsequently, 100 μl of cell suspension was inoculated subcutaneously into the dorsal root of the right hind limb in nude mice, and each nude mouse was inoculated with approximately 1 × 10^6^ tumor cells. Tumors were measured with vernier calipers every 3 days. The nude mice were killed under anesthesia after 6 weeks, and the skin was cut, followed by dissection of the intact transplanted tumors. The tumors were then weighed by electronic balance and the mass of terminal tumor was recorded.

### Immunohistochemistry

The microvessel density (MVD) in tumor tissues was measured in accordance with the Weidner criteria. Sections were observed under a low-power microscope. Five areas with the most stained microvessel were selected to search location rich in vessels, which were located in or near the tumor tissue area. Tumor tissues were collected for immunohistochemical staining, with the primary antibody against CD34 (ab81289, 1/2000, Abcam, Cambridge, MA, U.S.A.) used, and the vascular endothelial cells stained brown were considered as positive. MVD was counted under a high-power microscope according to the criteria for identifying any stained endothelial cells or cells as independent vessels. Five different visual fields were selected on each slide, and the stained vessels were simultaneously counted under a multi-eye fluoroscopy microscope to obtain the mean value.

### Statistical analysis

The data in the present research were analyzed by SPSS 21 (IBM Corp. Armonk, NY, U.S.A.). The measurement data were presented in the form of the mean ± standard deviation. First, the normality and the homogeneity of variance were tested. If the data were in accordance to the normal distribution and homogeneity of variance, intra-group comparison was conducted using paired *t*-test, inter-group comparison using unpaired *t-*test and data among multiple groups were compared by one-way analysis of variance (ANOVA) or repeated measurement ANOVA, and pairwise comparison by the post-hoc test. The data with skewed distribution or unequal variances were analyzed using the rank sum test.

## Results

### miR-613 influences the development of NPC via the AKT signaling pathway by regulating FN1

Four NPC-related microarray data GSE13597, GSE12452, GSE53819, and GSE64634 were retrieved from the GEO database. Differential analysis concerning the NPC samples and normal control samples in these four microarray data was conducted, obtaining 602, 766, 478, and 1033 DEGs, respectively. The heat maps of top 50 DEGs in four microarray data are shown in Figure 1A–D. Venn analysis of the four microarray data was conducted to further obtain DEGs in NPC (Figure 1E), revealing that 22 genes existed in the intersection of the four microarray data, which were all differentially expressed in the four NPC-related microarray data. The interaction among the 22 genes was further analyzed and the gene interaction network was constructed (Figure 1F), showing that FN1 gene was in the core of the 22 genes. Through the Kyoto Encyclopedia of Genes and Genomes (KEGG) database, FN1 gene was found to be located in the upstream of the AKT signaling pathway (map05205). Besides, the AKT signaling pathway has been reported to act an essential role in NPC [19,20], suggesting that FN1 might regulate NPC through the AKT signaling pathway. In order to further understand the upstream regulatory mechanism of FN1, the upstream regulatory miR of FN1 was predicted in databases such as DIANA, and the intersection of the predicted results was obtained (Figure 1G). Finally, six potential miRs regulating FN1 were obtained from the intersection, among which miR-613 was rarely studied in cancers, especially in NPC. Nevertheless, the other five miRs have already been reported in cancers including NPC [21–23]. Taken together, miR-613 participated in the development of NPC via the AKT signaling pathway by mediating the expression of FN1 gene. Then, miR-613 and FN1 expression in CNE1, CNE2, HONE1, 5-8F, and NP69 cell lines were measured by RT-qPCR and Western blot analysis (Figure 1H,I). In comparison with the NP69 cell line, the NPC cell lines exhibited significantly decreased miR-613 expression and obviously increased FN1 expression, of which HONE1 and CNE1 exhibited the relatively lower miR-613 expression but the relatively higher FN1 expression. Therefore, HONE1 and CNE1 cells were selected for follow-up experiment.

The article "microRNA-613 exerts anti-angiogenic effect on nasopharyngeal carcinoma cells through inactivating the AKT signaling pathway by down-regulating FN1" was retracted in 2021. Reasons: duplicated images; signs of a paper mill.

**Figure 1:** miR-613 participates in the development of NPC via the AKT signaling pathway by meditating FN1 (**A**–**D**) The heat maps of top 50 DEGs in NPC microarray data, in which the abscissa represented the sample number, the ordinate represented the gene name, and the left dendrogram showed clustering of the gene expression. Each small square referred to the expression of a gene in a sample; (**E**) Venn analysis of DEGs in NPC microarray data. Four ellipses in the diagram represented the DEGs of four different NPC microarray data, and the middle part represented the intersection of the results of four microarray data; (**F**) the gene interaction network for 22 genes in intersection of four microarray data; (**G**) prediction of miRs regulating FN1. Six triangles in the figure represented the predicted results in the six databases, and the middle part referred to the intersection of the predicted results; (**H**) relative expression of miR-613 and FN1 in NP69, CNE1, CNE2, HONE1, and 5-8F cell lines; *P < 0.05 compared with NP69 cell line. (**I**) The protein level of FNI examined by Western blot analysis. The measurement data were expressed as the mean ± standard deviation; data between two groups were compared by the paired *t-*test; data among multiple groups were compared by one-way ANOVA; the experiment was repeated three times.

### FN1 is the target gene of miR-613

The Target Scan website showed that a binding relationship between miR-613 and FN1 (Figure 2A). On this basis, dual luciferase reporter gene assay was conducted to verify the target relationship between miR-613 and FN1, and the results illustrated that compared with the NC group, the luciferase activity in FN1-Wt was obviously decreased (*P*<0.05) but that in FN1-Mut was not affected (*P*>0.05) with the overexpression of miR-613 (Figure 2B).

**Figure 2:** FN1 is the target gene of miR-613 (**A**) Binding site of miR-613 to FN1 in Target Scan website; (**B**) luciferase activity in FN1-Wt and FN1-Mut after transfection with miR-613 mimic; * *P*<0.05 compared with the NC group; (**C**) gray value of FN1 protein bands after alteration of miR-613 and FN1 in CNE1 cell; (**D**) protein expression of FN1 after transduction with miR-613 and FN1 in CNE1 cell; (**E**) gray value of FN1 protein bands after treatments with miR-613 and FN1 in HONE1 cell; (**F**) protein expression of FN1 after treatments with miR-613 and FN1 in HONE1 cell. *P<0.05 compared with the NC-mimic group; ^#^*P*<0.05 compared with the si-NC group; the measurement data were expressed as the mean ± standard deviation; data between two groups were compared by the unpaired *t*-test; data among multiple groups were compared by one-way ANOVA; the experiment was repeated three times; Wt, wild type; Mut, mutant type.

At the same time, protein expression of FN1 in HONE1 and CNE1 cell lines transfected with miR-613 mimic or si-FNI was detected by Western blot analysis. The results in CNE1 cell line revealed that compared with the blank group, the protein expression of FN1 did not differ in the NC-mimic group and the si-NC group (*P*>0.05). The protein expression of FN1 was greatly lower in the miR-613 mimic group than that in the NC-mimic group (*P*<0.05). Compared with the si-NC group, the si-FN1 group showed marked declines in protein expression of FN1 (*P*<0.05, Figure 2C,D). The results in HONE1 cell line were consistent with the results of CNE1 cell line (Figure 2E,F). These results suggested that miR-613 could target and down-regulate FN1.

The article "microRNA-613 exerts anti-angiogenic effect on nasopharyngeal carcinoma cells through inactivating the AKT signaling pathway by down-regulating FN1" was retracted in 2021. Reasons: duplicated images; signs of a paper mill.

### Overexpressed miR-613 or silenced FN1 represses cell proliferation, invasion, and migration, and promotes apoptosis in NPC by inactivating the AKT signaling pathway

Results of EdU assay for the detection of cell proliferation of HONE1 and CNE1 cells after transfection showed that compared with the blank group, there was no obvious difference in cell proliferation in the NC-mimic group and si-NC group (*P*>0.05), but cell proliferation was significantly reduced in the LY294002 group (*P*<0.05). Cell proliferation of the miR-613 mimic group was evidently inhibited versus that in the NC-mimic group (*P*<0.05). Relative to the si-NC group, the si-FN1 group exhibited dramatically suppressed cell proliferation (*P*<0.05). In comparison with miR-613 mimic-treated cells, proliferation was promoted in cells transfected with both miR-613 mimic and oe-FN1 (*P*<0.05, Figures 3A and 4A). Taken together, overexpression of miR-613, silencing of FN1 or LY294002 treatment had inhibitory effects on proliferation of NPC cells.

**Figure 3:** Up-regulated miR-613 or down-regulated FN1 contributes to suppressed cell proliferation, invasion, and migration, and promoted cell apoptosis of HONE1 cells (**A**) Cell proliferation of HONE1 cells after treatments with the mimic or inhibitor of miR-613 and FN1 as well as the LY294002 treatment detected by EdU (200×); (**B**) cell apoptosis of HONE1 cells after treatments with the mimic or inhibitor of miR-613 and FN1 as well as the LY294002 treatment examined by flow cytometry; (**C**) the protein bands of Bcl-2, Bax, Cleaved-caspase3 in HONE1 cells examined by Western blot analysis; (**D**) cell migration of HONE1 cells after treatments with the mimic or inhibitor of miR-613 and FN1 as well as the LY294002 treatment detected by Transwell assay (200×); (**E**) cell invasion of HONE1 cells after treatments with the mimic or inhibitor of miR-613 and FN1 as well as the LY294002 treatment detected by Transwell assay (200×); (**F**) protein expression of MMP-2 and MMP-9 in HONE1 cells after treatments with the mimic or inhibitor of miR-613 and FN1 as well as the LY294002 treatment examined by Western blot analysis. ^&^*P*<0.05 compared with the blank group; *P<0.05 compared with the NC mimic group; ^#^*P*<0.05 compared with the si-NC group; ^@^*P*<0.05 compared with the miR-613 mimic group; the measurement data were expressed as the mean ± standard deviation; data among multiple groups were compared by one-way ANOVA; the experiment was repeated three times.

The article "microRNA-613 exerts anti-angiogenic effect on nasopharyngeal carcinoma cells through inactivating the AKT signaling pathway by down-regulating FN1" was retracted in 2021. Reasons: duplicated images; signs of a paper mill.

**Figure 4:** Up-regulated miR-613 or down-regulated FN1 contributes to suppressed cell proliferation, invasion, and migration, and promoted cell apoptosis of CNE1 cells (**A**) Cell proliferation of CNE1 cells after treatments with the mimic or inhibitor of miR-613 and FN1 as well as the LY294002 treatment detected by EdU (200×); (**B**) cell apoptosis of CNE1 cells after treatments with the mimic or inhibitor of miR-613 and FN1 as well as the LY294002 treatment examined by flow cytometry; (**C**) the protein bands of Bcl-2, Bax, Cleaved-caspase3 in CNE1 cells examined by Western blot analysis; (**D**) cell migration of CNE1 cells after treatments with the mimic or inhibitor of miR-613 and FN1 as well as the LY294002 treatment detected by Transwell assay (200×); (**E**) cell invasion of CNE1 cells after treatments with the mimic or inhibitor of miR-613 and FN1 as well as the LY294002 treatment detected by Transwell assay (200×); (**F**) protein expression of MMP-2 and MMP-9 in CNE1 cells after treatments with the mimic or inhibitor of miR-613 and FN1 as well as the LY294002 treatment examined by Western blot analysis. ^&^*P*<0.05 compared with the blank group; *P<0.05 compared with the NC mimic group; ^#^*P*<0.05 compared with the si-NC group; ^@^*P*<0.05 compared with the miR-613 mimic group; the measurement data were expressed as the mean ± standard deviation; data among multiple groups were compared by one-way ANOVA; the experiment was repeated three times.

Results of flow cytometry, which was performed to assess cell apoptosis of HONE1 and CNE1 cells after transfection, showed that the apoptosis rate did not differ greatly in the NC-mimic group and the si-NC group compared with blank group (*P*>0.05). However, in contrast to the blank group, the LY294002 group presented obviously increased apoptosis rate of NPC cells (*P*<0.05). Compared with the NC-mimic group, the apoptosis rate of NPC cells in the miR-613 mimic group was significantly elevated (*P*<0.05). Compared with the si-NC group, the apoptosis rate of NPC cells in the si-FN1 group was greatly increased (*P*<0.05). In comparison with the NPC cells treated with miR-613 mimic, the NPC cells treated with both miR-613 mimic and oe-FN1 displayed down-regulated apoptosis rate (*P*<0.05, Figures 3B and 4B). These findings demonstrated that miR-613 overexpression, FN1 silencing, or LY294002 treatment could promote apoptosis of NPC cells.

Subsequently, Western blot analysis was applied to examine the protein expression of proliferation-related factors and apoptosis-related factors in HONE1 and CNE1 cells. It revealed that in comparison with the blank group, the NC-mimic and si-NC groups showed no significant difference in the expression of Bcl-2, Bax, and Cleaved-caspase3 (*P*>0.05), while the LY294002 group exhibited significantly lower ratio of Bcl-2/Bax but obviously higher expression of Cleaved-caspase3 (*P*<0.05). In contrast to the NC-mimic group, significantly decreased ratio of Bcl-2/Bax and obviously increased expression of Cleaved-caspase3 were found in the miR-613 mimic group (*P*<0.05). Compared with the si-NC group, the si-FN1 group depicted lower ratio of Bcl-2/Bax but higher expression of Cleaved-caspase3 (*P*<0.05). Besides, obviously increased ratio of Bcl-2/Bax and decreased expression of Cleaved-caspase3 were found after co-treatment with miR-613 mimic and oe-FN1 compared with the miR-613 mimic treatment alone (*P*<0.05, Figures 3C and 4C). From these findings, a conclusion could be drawn that miR-613 overexpression, FN1 silencing, or LY294002 treatment decreased the ratio of Bcl-2/Bax and increased expression of Cleaved-caspase3.

The article "microRNA-613 exerts anti-angiogenic effect on nasopharyngeal carcinoma cells through inactivating the AKT signaling pathway by down-regulating FN1" was retracted in 2021. Reasons: duplicated images; signs of a paper mill.

Transwell assay was performed for detection of cell migration and invasion of HONE1 and CNE1 cells after transfection. The results suggested that versus the blank group, there was no evident difference concerning the migration and invasion of cells in the NC-mimic group and the si-NC group (*P*>0.05) while cell migration and invasion were significantly attenuated in the LY294002 group (*P*<0.05). Compared with the NC-mimic group, the miR-613 mimic group exhibited inhibited cell migration and invasion (*P*<0.05). Cell migration and invasion in the si-FN1 group were markedly attenuated in contrast to that in the si-NC group (*P*<0.05). Compared with the NPC cells treated with miR-613 mimic, the migration and invasion in NPC cells transfected with miR-613 mimic and oe-FN1 were dramatically promoted (*P*<0.05, Figures 3D and 4D). Therefore, miR-613 elevation, FN1 down-regulation or LY294002 treatment inhibited cell migration and invasion in NPC.

Here, the levels of factors related to migration (Figures 3E and 4E) and invasion in HONE1 and CNE1 cells after transfection was measured by Western blot analysis. It revealed that the levels of MMP-2 and MMP-9 in the NC-mimic and si-NC groups were not remarkably different from those in the blank group (*P*>0.05), but the expression of MMP-2 and MMP-9 in the LY294002 group was evidently down-regulated versus the blank group (*P*<0.05). Compared with the NC-mimic group, the expression of MMP-2 and MMP-9 in the miR-613 mimic group was greatly decreased (*P*<0.05). The si-FN1 group presented evident declines in the expression of MMP-2 and MMP-9, relative to the si-NC group (*P*<0.05). In comparison with the miR-613 mimic group, the expression of MMP-2 and MMP-9 in the miR-613 mimic + oe-FN1 group was greatly up-regulated (*P*<0.05, Figures 3F and 4F). From these results, the conclusion could be made that overexpressed miR-613, silenced FN1 or the LY294002 treatment could lead to suppressed migration and invasion of NPC cells.

The article "microRNA-613 exerts anti-angiogenic effect on nasopharyngeal carcinoma cells through inactivating the AKT signaling pathway by down-regulating FN1" was retracted in 2021. Reasons: duplicated images; signs of a paper mill.

### Overexpression of miR-613 or silencing of FN1 inhibits angiogenesis of NPC cells

The results of tube formation assay, which was employed to assess angiogenesis of HONE1 and CNE1 cells after transfection, suggested that the angiogenesis rate did not differ in the NC-mimic group and the si-NC group compared with the blank group (*P*>0.05). However, the LY294002 group exhibited a significant decline in angiogenesis rate in comparison with the blank group (*P*<0.05). NPC cells transfected with miR-613 mimics showed obviously reduced angiogenesis rate versus cells transfected with NC-mimic (*P*<0.05). Compared with the si-NC group, the angiogenesis rate of the si-FN1 group was significantly decreased (*P*<0.05). Relative to the miR-613 mimic group, the miR-613 mimic + oe-FN1 group exhibited obviously enhanced angiogenesis rate (*P*<0.05, Figure 5A,B). Thus, a conclusion could be made that overexpression of miR-613, silencing of FN1 or LY294002 treatment exerted inhibitory effects on angiogenesis of NPC cells by inactivating the AKT signaling pathway.

**Figure 5:** Angiogenesis of NPC cells is suppressed with the overexpression of miR-613 or silencing of FN1 (**A**) Angiogenesis ability of CNE1 cells after treatments with the mimic or inhibitor of miR-613 and FN1 as well as the LY294002 treatment detected by tube formation assay (100×); (**B**) angiogenesis ability of HONE1 cells after treatments with the mimic or inhibitor of miR-613 and FN1 as well as the LY294002 treatment detected by tube formation assay (100×); (**C**) protein expression of angiogenesis-related factors (VEGF and CD31) in CNE1 cells after treatments with the mimic or inhibitor of miR-613 and FN1 as well as the LY294002 treatment examined by Western blot analysis; (**D**) protein expression of angiogenesis-related factors (VEGF and CD31) in HONE1 cells after treatments with the mimic or inhibitor of miR-613 and FN1 as well as the LY294002 treatment detected by Western blot analysis. ^&^*P*<0.05 compared with the blank group; *P<0.05 compared with the NC mimic group; ^#^*P*<0.05 compared with the si-NC group; ^@^*P*<0.05 compared with the miR-613 mimic group; the measurement data were expressed as the mean ± standard deviation; data among multiple groups were compared by one-way ANOVA; the experiment was repeated three times.

Expression of angiogenesis-related factors VEGF and CD31 in HONE1 and CNE1 cells after transfection was measured by Western blot analysis. The results showed that the expression of VEGF and CD31 did not differ in the NC-mimic group and the si-NC group in comparison with the blank group (*P*>0.05), but the levels of VEGF and CD31 were significantly reduced in the LY294002 group (*P*<0.05). The expression of VEGF and CD31 was greatly down-regulated in the miR-613 mimic group (*P*<0.05) compared with the NC-mimic group, reduced in the si-FN1 group versus the si-NC group (*P*<0.05), and elevated in miR-613 mimic + oe-FN1 group relative to the miR-613 mimic group (*P*<0.05, Figure 5C,D). Taken together, the levels of angiogenic factors were decreased due to the overexpression of miR-613, silencing of FN1 or LY294002 treatment.

The article "microRNA-613 exerts anti-angiogenic effect on nasopharyngeal carcinoma cells through inactivating the AKT signaling pathway by down-regulating FN1" was retracted in 2021. Reasons: duplicated images; signs of a paper mill.

### miR-613 inactivate the AKT signaling pathway through inhibiting FN1 in NPC

In order to determine the effects of miR-613 on the AKT signaling pathway, HONE1 and CNE1 cells were transfected with miR-613 overexpression or FN1 silencing to conduct Western blot analysis for the determination of the protein expression of factors related to the AKT signaling pathway protein and phosphorylated proteins. Compared with the blank group, there was no significant difference in the expression of AKT and mTOR as well as the phosphorylation extents of AKT and mTOR in the NC-mimic group and the si-NC group (*P*>0.05). In the LY294002 group, AKT and mTOR expression and their phosphorylation extents were remarkably inhibited versus the blank group (*P*<0.05). Compared with the NC-mimic group, the expression and phosphorylation extents of AKT and mTOR were significantly down-regulated in the miR-613 mimic group (*P*<0.05). The si-FN1 group exhibited evident declines in expression and phosphorylation extents of AKT and mTOR, relative to the si-NC group (*P*<0.05). Compared with the miR-613 mimic group, the expression and phosphorylation extents of AKT and mTOR in the miR-613 mimic + oe-FN1 group were significantly up-regulated (*P*<0.05, Figure 6A–D). Hence, overexpression of miR-613 down-regulated FN1, thus inactivating the AKT signaling pathway.

**Figure 6:** miR-613 overexpression leads to inactivation of the AKT signaling pathway via down-regulation of FN1 (**A**) Gray value of AKT, mTOR, p-AKT, and p-mTOR protein bands in CNE1 cells examined by Western blot analysis; (**B**) protein expression and phosphorylation extents of AKT and mTOR in CNE1 cells; (**C**) gray value of AKT, mTOR, p-AKT, and p-mTOR protein bands in HONE1 cells examined by Western blot analysis; (**D**) protein expression and phosphorylation extents of AKT and mTOR in HONE1 cells. ^&^*P*<0.05 compared with the blank group; *P<0.05 compared with the NC mimic group; ^#^*P*<0.05 compared with the si-NC group; ^@^*P*<0.05 compared with the miR-613 mimic group; the measurement data were expressed as the mean ± standard deviation; data among multiple groups were compared by one-way ANOVA; the experiment was repeated three times.

The article "microRNA-613 exerts anti-angiogenic effect on nasopharyngeal carcinoma cells through inactivating the AKT signaling pathway by down-regulating FN1" was retracted in 2021. Reasons: duplicated images; signs of a paper mill.

### Overexpression of miR-613 or silencing of FN1 inhibits tumorigenesis and angiogenesis

Tumorigenic ability and neovascular MVD in HONE1 cell after transfection were detected by xenograft in nude mice and immunohistochemistry, respectively. The results suggested that in comparison with the blank group, tumor growth rate, tumor weight, and MVD did not differ in the NC-mimic group and the si-NC group (all *P*>0.05) but the tumor growth rate, tumor weight and MVD were significantly reduced in the LY294002 group (*P*<0.05). Mice in the miR-613 mimic group exhibited lower tumor growth rate, tumor weight, and MVD, relative to mice in the NC-mimic (*P*<0.05). In comparison with the si-NC group, the tumor growth rate, tumor weight, and MVD were significantly decreased in the si-FN1 group (*P*<0.05). In contrast to the miR-613 mimic group, the tumor growth rate, tumor weight, and MVD were significantly elevated in the miR-613 mimic + oe-FN1 group (*P*<0.05, Figure 7A–E). The results demonstrated that overexpression of miR-613, silencing of FN1, or LY294002 treatment could inhibit the tumorigenesis and angiogenesis.

**Figure 7:** miR-613 up-regulation or FN1 down-regulation leads to repressed tumorigenesis and angiogenesis in nude mice (**A**) Tumor volume of nude mice after transfection; (**B**) tumor weight growth curve of nude mice; (**C**) tumor weight of nude mice; (**D**) MVD of xenograft examined by immunohistochemistry (400×); (**E**) the histogram of MVD in tumors. ^&^*P*<0.05 compared with the blank group; *P<0.05 compared with the NC mimic group; ^#^*P*<0.05 compared with the si-NC group; ^@^*P*<0.05 compared with the miR-613 mimic group; the measurement data were expressed as mean ± standard deviation; data among multiple groups were compared by one-way ANOVA or repeated measure ANOVA.

## Discussion

NPC is a squamous cell carcinoma that derives from the nasopharynx epithelium, which presents remarkable geographical and racial differences [3,5]. Up to now, several EBV-encoded and human miRs have been evidenced to be dysregulated in NPC, thus exerting functions in the tumorigenesis, metastasis and invasion of NPC cells [1]. Nevertheless, the potential mechanism of miR-613 in NPC is still unclear, and the present study probes into a new potential role of miR-613, FN1, and AKT signaling pathway in modulating invasion, migration, and angiogenesis of NPC cells. As a consequence, the present study demonstrates that up-regulation of miR-613 suppresses NPC cell invasion, metastasis, and angiogenesis through inactivation of the AKT signaling pathway by inhibiting FN1.

The article "microRNA-613 exerts anti-angiogenic effect on nasopharyngeal carcinoma cells through inactivating the AKT signaling pathway by down-regulating FN1" was retracted in 2021. Reasons: duplicated images; signs of a paper mill.

Initially, our results demonstrated that down-regulation of miR-613 and overexpression of FN1 was found in NPC tissues. Similarly, Wang et al. found that miR-613 expression was remarkably reduced in HCC cells [10]. Results of the study conducted by Guan and his team indicated the down-regulation of miR-613 in serum samples and cancerous tissue of patients with esophageal squamous cell carcinoma [12]. Meanwhile, a previous study emphasized that up-regulation of miR-613 suppressed NPC cell invasion induced by Snail2 [11]. Previous studies found that FN1 expression is significantly high in NPC tissues and FN1 plays a crucial role in cell metastasis and differentiation [13,24].

Next, the results of dual luciferase reporter gene assay demonstrated that miR-613 could target FN1; miR-613 suppresses invasion, metastasis, and angiogenesis of NPC cells by targeting FN1. Overexpressed miR-613 has been revealed to inhibit the bladder cancer cell invasion, proliferation, and metastasis via regulation of the expression of Sphk1 [25], which was partly consistent with our results. Interestingly, a very recent study proved that up-regulation of miR-613 suppressed cell invasion, metastasis, and proliferation through directly targeting and inhibiting VEGFA [26]. Up-regulated miR-15a and miR-16 inhibited angiogenesis multiple myeloma by targeting VEGF, which was proved by a recent study [27]. Interestingly, overexpressed miR-92a in angiogenic endothelial cells was reported to exert an anti-angiogenic function in cancer [28]. Moreover, it is revealed that FN1 is a target gene of miR-613 [12]. FN1, a member of ECM glycoprotein family, plays a key role in cellular adhesion, migration polarity, and tissue remodeling; FN1 is also conducive to microvascular integrity maintenance and infection resistances [13]. Furthermore, it has been recently verified that FN1 was closely correlated to cell metastasis, differentiation, and adhesion in various cancers, and the down-regulation of FN1 causes suppression of the invasion and metastasis in cancer cells [24]. Consistently, FN1 down-regulation could repress cell invasion, metastasis, and proliferation in esophageal cancer cells [29]. Additionally, it was suggested that attenuated FN1 could effectively repress the metastasis of gastric cancer cells, and that miR-200c could lead to suppression of the invasion, metastasis, and proliferation of gastric cancer cells via the down-regulation of FN1 [30].

Besides, our research also revealed that overexpression of miR-613 reduces tumor invasion, metastasis, and angiogenesis in NPC through inactivating the AKT signaling pathway by inhibiting FN1. AKT signaling pathway acts an essential function in modulating several cellular processes, such as cell survival, proliferation, apoptosis, and nutrient metabolism, which function in both normal and cancer cells [31]. A previous study suggested that AKT signaling pathway played a key role in carcinogenesis of NPC, and that down-regulation of AKT signaling pathway suppressed the development of NPC cells [32]. In addition, suppressing the activation of AKT signaling pathway was demonstrated to inhibit invasion and metastasis in NPC cells [33]. miR-613 was demonstrated to influence I/R-induced cardiomyocyte apoptosis through regulating the AKT signaling pathway, reported by a very recent study by Wu et al. [16]. The results of the current study provide evidence that FN1 regulates NPC via the AKT signaling pathway.

The article "microRNA-613 exerts anti-angiogenic effect on nasopharyngeal carcinoma cells through inactivating the AKT signaling pathway by down-regulating FN1" was retracted in 2021. Reasons: duplicated images; signs of a paper mill.

## Conclusions

In line with the previous studies, we have confirmed down-regulation of miR-613 and overexpression of FN1 in NPC tissues. We also demonstrate that FN1 is the target gene of miR-613, and up-regulation of miR-613 suppresses invasion, migration, and angiogenesis in NPC cells through inactivation of AKT signaling pathway via down-regulation of FN1 (Figure 8). Therefore, we speculate that miR-613 may be potential new direction in the treatment of NPC. Nevertheless, further study is required to probe into the mechanism through which miR-613 regulates the AKT signaling pathway in the cancer.

**Figure 8:** Regulatory mechanism by which miR-613 mediated migration, invasion, and angiogenesis in NPC via the AKT signaling pathway by regulating FN1 miR-613 overexpression and FN1 silencing inactivated the AKT signaling pathway to inhibit invasion, migration, and angiogenesis in NPC, corresponding to down-regulated Bcl-2, MMP-2, MMP-9, VEGF, and CD31 as well as decreased the ratio of Bcl-2/Bax and increased expression of Cleaved-caspase3.

## Abbreviations

ANOVA: analysis of variance
Bax: Bcl-2-associated X protein
Bcl_2_: B-cell lymphoma 2
CD31: cell adhesion molecule-1
DEG: differentially expressed gene
EBV: Epstein–Barr virus
EdU: 5-ethynyl-2′-deoxyuridine
FN1: Fibronectin 1
GAPDH: glyceraldehyde-3-phosphate dehydrogenase
GEO: Gene Expression Omnibus
HCC: hepatocellular carcinoma
miR-613: microRNA-613
MMP: matrix metallopeptidase
mTOR: mammalian target of rapamycin
MVD: microvessel density
NC: negative control
NPC: nasopharyngeal carcinoma
RT-qPCR: reverse transcription quantitative polymerase chain reaction
VEGF: vascular endothelial growth factor
